# The Emerging Role of Estrogens in Thyroid Redox Homeostasis and Carcinogenesis

**DOI:** 10.1155/2019/2514312

**Published:** 2019-01-09

**Authors:** Caroline C. Faria, Milena S. Peixoto, Denise P. Carvalho, Rodrigo S. Fortunato

**Affiliations:** ^1^Laboratório de Fisiologia e Sinalização Redox, Instituto de Biofísica Carlos Chagas Filho, Universidade Federal do Rio de Janeiro, Rio de Janeiro 21941-902, Brazil; ^2^Laboratório de Fisiologia Endócrina Doris Rosenthal, Instituto de Biofísica Carlos Chagas Filho, Universidade Federal do Rio de Janeiro, Rio de Janeiro 21941-902, Brazil

## Abstract

Reactive oxygen species (ROS) are the most critical class of free radicals or reactive metabolites produced by all living organisms. ROS regulate several cellular functions through redox-dependent mechanisms, including proliferation, differentiation, hormone synthesis, and stress defense response. However, ROS overproduction or lack of appropriate detoxification is harmful to cells and can be linked to the development of several diseases, such as cancer. Oxidative damage in cellular components, especially in DNA, can promote the malignant transformation that has already been described in thyroid tissue. In thyrocyte physiology, NADPH oxidase enzymes produce large amounts of ROS that are necessary for hormone biosynthesis and might contribute to the high spontaneous mutation rate found in this tissue. Thyroid cancer is the most common endocrine malignancy, and its incidence is significantly higher in women than in men. Several lines of evidence suggest the sex hormone estrogen as a risk factor for thyroid cancer development. Estrogen in turn, besides being a potent growth factor for both normal and tumor thyroid cells, regulates different mechanisms of ROS generation. Our group demonstrated that the thyroid gland of adult female rats exhibits higher hydrogen peroxide (H_2_O_2_) production and lower enzymatic antioxidant defense in comparison with male glands. In this review, we discuss the possible involvement of thyroid redox homeostasis and estrogen in the development of thyroid carcinogenesis.

## 1. Introduction

The maintenance of cellular redox homeostasis is essential for a correct cellular function; therefore, the cells must keep an appropriate balance between oxidative and antioxidant mechanisms. Reactive oxygen species (ROS) are common by-products of the aerobic cellular metabolism, being continuously formed in the cells. ROS include the superoxide anion (O_2_^•−^), hydrogen peroxide (H_2_O_2_), and hydroxyl radicals (OH^•^), among others, all of which have inherent chemical properties that confer reactivity to different biological targets [1, 2].

The formation of ROS can occur through enzymatic or nonenzymatic reactions and under the influence of endogenous or exogenous factors. Cellular ROS are produced by the mitochondrial respiratory chain and also by enzyme-catalyzed reactions involving NADPH oxidases (NOX), xanthine oxidase, nitric oxide synthase (NOS), cytochrome P450 enzymes, lipoxygenase, and cyclooxygenase [3, 4]. The maintenance of intracellular redox homeostasis is also dependent on a complex set of antioxidant molecules. These antioxidants include low molecular weight molecules, such as glutathione (GSH) that is present at millimolar concentrations within cells, as well as alpha-lipoic acid, coenzyme Q, ferritin, uric acid, bilirubin, metallothionein, l-carnitine, melatonin, and also a wide range of antioxidant proteins that have a specific subcellular localization and chemical reactivities (e.g., superoxide dismutase (SOD), catalase (CAT), glutathione peroxidase (GPX), glutathione reductase (GR), thioredoxin reductase (TRX), and peroxiredoxins (PRXs)) [2].

Oxidative stress is characterized by a prooxidant environment that results from the imbalance between ROS production and elimination. Several studies suggest an important role of ROS in the pathophysiology of a wide range of diseases, since these molecules have the ability to react and damage cellular constituents, such as lipids, proteins, and DNA [5]. Indeed, oxidative stress occurs not only when irreversible oxidative damage or a widespread prooxidant status is established in the cell but also when any change in the mechanism of production and/or degradation of ROS disrupts the normal functioning of cell redox-sensitive systems [6]. In this context, in the past two decades, it has become apparent that ROS also act as signaling molecules to regulate biological and physiological processes [7].

The primary function of the thyroid gland is to synthesize the thyroid hormones (THs) L-3,5,3′,5′-tetraiodothyronine (T4) and L-3,5,3′-triiodothyronine (T3). The follicular thyroid cells uptake iodide from blood circulation and incorporate it into thyroglobulin (Tg), the precursor of TH. Iodide oxidation, iodination of tyrosyl residues in the Tg molecule, and the coupling of iodotyrosines are all steps of TH biosynthesis catalyzed by thyroperoxidase (TPO), which requires high concentrations of H_2_O_2_ as cosubstrate. In this case, the source of H_2_O_2_ is specifically dual oxidase 2 enzyme (DUOX2), a member of the NOX family [8]. Besides having a crucial role in TH synthesis, H_2_O_2_ can be toxic for thyrocytes, as it is a mutagenic and carcinogenic molecule [9].

The prevalence of thyroid cancer is described in the literature to be about 3-4 times higher in women than in men worldwide [10]. While in prepubertal individuals thyroid cancer is rare and approximately invariable, with the advent of puberty, the incidence becomes 14 times higher, reaching the peak age of incidence during the reproductive period in females [11, 12]. In addition, after menopause, the incidence decreases again [13]. Albeit genetic alterations (*BRAF*, *RAS*, and *RET* mutations), ionizing radiation exposure and iodine deficiency are the main triggers for thyroid cancer pathogenesis; these mechanisms do not seem to be related to this gender disparity [10]. Thus, the scientific community has recognized a remarkable role for sex hormones, especially estrogens, in the development of thyroid cancer [14, 15].

Indeed, some studies have reported that prolonged exposure to exogenous estrogens is linked to thyroid cancer [16–18]. Other studies have pointed to an increased risk of this disease in women who had been treated with estrogens for gynecological disorders or taking oral contraceptives [19]. Early menarche, a higher number of ovulatory cycles, and pregnancies have also been correlated with higher thyroid cancer incidence [20, 21]. A more recent prospective study showed that hormone replacement therapy with estrogen monotherapy, but not progestin monotherapy or progestin combined with estrogen, was notably associated with increased risk of thyroid cancer [22]. Despite these consistent findings that show a strong influence of estrogen in thyroid carcinogenesis, the molecular mechanisms underlying estrogens' deleterious effects on the thyroid remain to be clarified. Interestingly, estrogen increases ROS generation that can culminate in cancer initiation, as well as promotion and progression. In the present review, we will focus on the influence of ROS in thyroid carcinogenesis and the contribution of estrogen in the disruption of thyroid redox homeostasis that could explain the sexual dimorphism found in thyroid cancer.

## 2. Redox Homeostasis and Signaling

The availability of ROS in a given site results from the balance between its production, from various sources, and its disposal, by enzymatic and nonenzymatic antioxidants. The most relevant source of ROS is due to the incomplete reduction of molecular oxygen used to drive the mitochondrial respiratory chain or is related to the activity of NOX in biological membranes, generating superoxide or H_2_O_2_ [23]. Superoxide is rapidly converted into H_2_O_2_ spontaneously or by the enzymatic reaction catalyzed by superoxide dismutase (SOD). While SOD1 is primarily located in the cytosol, SOD2 localizes to the mitochondrial matrix and SOD3 seems to be in the extracellular compartment. These enzymes prevent the accumulation of superoxide, which is extremely reactive and can damage proteins [24]. Besides, the relatively stable nature of H_2_O_2_ makes it suitable to act as a second messenger in redox signaling [25]. Hydroxyl radical, in turn, is extremely reactive and can oxidize lipids, proteins, and DNA indiscriminately, resulting in damage to these macromolecules and so triggering cellular stress. Typically, hydroxyl radicals are generated from H_2_O_2_ in the presence of ferrous ions (i.e., the Fenton reaction). Therefore, cells have multiple mechanisms to maintain iron homeostasis and prevent the formation of toxic hydroxyl radicals [26].

Production of ROS can be counterbalanced by multiple antioxidant systems. Peroxiredoxins (PRXs) are the most abundant intracellular antioxidant proteins that belong to a ubiquitous family of enzymes that share the same basic catalytic mechanism, in which an active-site cysteine (the peroxidatic cysteine) is oxidized to a cysteine sulfenic acid by a peroxide substrate [27]. TRX is a small protein containing two adjacent thiol groups in its reduced form, which are converted to a disulfide unit when oxidized. The reduction of the disulfide unit back to the dithiol form is catalyzed by the thioredoxin reductase (TR), using NADPH as an electron donor [28]. The heme enzyme catalase acts by converting H_2_O_2_ into water and molecular oxygen and is localized mainly in peroxisomes. Moreover, cells produce a large pool of GSH, which can be oxidized to glutathione disulfide (GSSG), independently, or catalyzed by glutathione peroxidases (GPX). Reduction of GSSG to GSH is catalyzed by glutathione reductases (GR) in a NADPH-dependent reaction. It is important to note that the variations in H_2_O_2_ required for signaling do not cause significant changes in the intracellular ratio of GSSG/GSH. It does not affect the ratio of NADPH to its oxidized form, NADP^+^, utilized to regenerate a myriad of antioxidants, including glutathione [29]. Large changes in these parameters are usually a sign of oxidative stress causing toxicity rather than signaling cascades associated with redox biology [28].

At low or moderate levels, ROS can act as signaling molecules sustaining cellular proliferation and differentiation and activating stress responsive survival pathways [30]. For instance, through inhibition of phosphatases, ROS can activate a wide range of signaling molecules, such as protein kinase C (PKC), p38 mitogen-activated protein kinase (p38 MAPK), extracellular signal-regulated kinase 1/2 (ERK1/2), phosphoinositide 3-kinase/serine-threonine kinase (PI3K/Akt), protein kinase B (PKB), and JUN N-terminal kinase (JNK) [31–33]. In addition, ROS are able to induce the expression of antioxidant genes via activation of the nuclear factor erythroid 2-related factor 2 (Nrf2). Nrf2 binds to antioxidant response elements (ARE), a specific sequence present in the promoter regions of the target genes, as a heterodimer with a small Maf protein, and stimulates the transcription of antioxidant proteins, such as glutathione-S-transferase (GST) and NADPH:quinone oxidoreductase 1 (NQO1), among others [34]. ROS are also involved in the activation of other transcription factors, such as activator protein 1 (AP-1), nuclear factor-*κ*B (NF-*κ*B), hypoxia-inducible transcription factor 1*α* (HIF-1*α*), and p53 [35, 36], all of them related with antioxidant responses.

Redox signaling occurs mainly through H_2_O_2_-mediated oxidation of the thiolate side chain of cysteine residues within proteins [37]. Cysteine oxidation can directly influence enzyme activity or act as a linker to form complexes with other redox-sensitive proteins through disulfide bridges, altering the activity of signaling pathways [38]. H_2_O_2_ is able to oxidize thiolate anion (Cys-S-) from cysteine residues to a sulfenic form (Cys-SOH), causing allosteric modifications that can be reversed by thioredoxin reductase (TR) and glutaredoxin (GRX), which turn the protein into its original state. Therefore, this structural change serves as a reversible signal transduction mechanism at physiological levels of H_2_O_2_. Nevertheless, higher levels of H_2_O_2_ further oxidize thiolate anions to sulfinic (SO_2_H) or sulfonic (SO_3_H) species. Unlike sulfenic modifications, sulfinic and sulfonic modifications are irreversible and result in permanent protein damage [39].

Redox signaling can vary within different organelles and cell compartments, depending on the presence of ROS generating and detoxifying systems, which ensure specificity to redox signaling. The H_2_O_2_-dependent oxidation of a given protein is likely to occur close to the source of H_2_O_2_ production. For example, the targets of H_2_O_2_ generated by NADPH oxidases present at the plasma membrane are probably also located nearby. Mitochondria are known to move dynamically towards their targets, thus allowing mitochondrion-generated H_2_O_2_ to activate specific signaling pathways [40]. Similarly, superoxide accumulation in the mitochondrial matrix has different outcomes from superoxide accumulation in the cytosol, in part due to a high content of iron-sulfur cluster proteins in the mitochondrial matrix [41].

Finally, the ataxia-telangiectasia-mutated (ATM) protein kinase, which is best known for its role in the DNA damage response, was found to function as a redox sensor, controlling the levels of ROS in human cells [42]. It was demonstrated that hematopoietic stem cells from ATM-null mice have higher ROS levels that activate p38 MAPK, resulting in a reduction of the repopulating capacity of these stem cells [43]. In fact, the antioxidant N-acetylcysteine (NAC) rescues some of the defects that result from the loss of ATM, suggesting that the normal function of ATM might be to control ROS levels [44, 45]. When ATM is classically activated by double-strand DNA breaks, the protein undergoes monomerization and requires free DNA ends and the Mre11-Rad50-Nbs1 (MRN) complex. By contrast, oxidized ATM is an active dimer in which the two monomers are covalently linked by intermolecular disulfide bonds that promote antioxidant responses [46, 47]. These observations emphasize the importance of ATM as a tumor suppressor, both due to its role in the DNA damage response, as well as to its effects on redox homeostasis.

## 3. Redox Homeostasis and Carcinogenesis

Carcinogenesis is a multifactorial and multistep process that is didactically described by three stages: initiation, marked by the acquisition of irreversible modifications in DNA, such as point mutations or chromosomal aberrations; promotion, characterized by shifts on cellular dynamics as a result of exogenous or endogenous molecules that interfere in cell proliferation, cell death, inflammation, and gene expression; and progression, driven by increased motility, invasiveness, and angiogenesis [48, 49]. In this context, high ROS availability can induce from DNA damage that leads to genomic instability and contributes to cancer initiation to the constant activation of several transcription factors (e.g., NF-*κ*B, AP-1, and HIF-1), modifying the cell fates during tumor promotion and progression [50–52]. Thus, ROS are thought to play multiple roles in tumor establishment and maintenance (Figure 1).

Cancer cells show higher levels of ROS when compared to their normal counterparts. High endogenous levels of oxidative stress have been found in several types of leukemia [53], in human colorectal carcinoma [54], as well as in breast [55], stomach [56], and ovarian cancer [57]. Moreover, ROS levels in prostate cancer positively correlate with tumor aggressiveness [58]. The mechanisms underlying the disrupted redox homeostasis include hypoxia, enhanced cellular metabolic activity, mitochondrial dysfunction, oncogene activation, higher activity of oxidases, lipoxygenases, and cyclooxygenases, and the crosstalk between cancer and immune cells recruited to the tumor site. On the other hand, the recent studies revealed that neoplastic cells are able to develop powerful antioxidant mechanisms to counterbalance excessive ROS, maintaining their redox status compatible with survival and thus suppressing apoptosis [59, 60]. This phenomenon may be a consequence of cellular adaptation and could play an important role in the development of malignant behavior and drug resistance [61].

ROS can interact with DNA causing a range of alterations, such as apurinic/apyrimidinic DNA sites, oxidized purines and pyrimidines, single- and double-strand DNA breaks (SSDs and DSBs), and DNA protein cross-linkages that cannot be repaired [62, 63]. In fact, increased levels of oxidative DNA lesions have been implicated in the etiopathology of various cancers. Hydroxyl radicals may interact with guanines giving rise to the two most common DNA base modifications: 8-oxo-7,8-dihydroguanine (8-oxodG) and 2,6-diamino-4-hydroxy-5-formamidopyrimidine (FapydG). Both alterations arise from the addition of the hydroxyl radical to the C8 position of the guanine ring, producing the 8-hydroxy-7,8-dihydroguanyl radical that can be oxidized into 8-oxodG or reduced to FapydG [64]. Furthermore, hydroxyl radical can also interact with pyrimidines, leading to the formation of 5,6-dihydroxy-5,6-dihydrothymine (thymine glycol) and 5,6-dihydroxy-5,6-dihydrocytosine (cytosine glycol) [62]. 8-oxodG and thymine glycol are the most studied DNA lesions that have been widely used as markers of oxidative stress. These DNA lesions are not necessarily lethal to the cell but are considered highly mutagenic, since in a given cell, about 10^5^ oxidative lesions occur per day [65]. The apurinic/apyrimidinic DNA sites are mainly formed as intermediates during the repair of oxidized bases and show a high mutagenic potential through the possible block of DNA polymerases [66]. The interaction of hydroxyl radicals with the deoxyribose backbone of DNA can lead to DNA SSBs and DSBs [62]. Besides, ROS-mediated mutations can also occur in mitochondrial DNA (mtDNA), mainly due to its close proximity to the respiratory chain, which leads to an increased probability of DNA damage by ROS. Moreover, mtDNA is not protected by histones, has high transcription rates, is intronless, and does not express DNA repair enzymes [67, 68]. As a result, nuclear repair enzymes need to be translocated into the mitochondria that also lack the nucleotide excision repair (NER) mechanism.

High levels of ROS might also cause direct protein damage, triggering conformational changes that are related to alterations in its function (gain of function, loss of function, or switch to a different function). Changes in protein tridimensional conformation affect its binding capacity to other proteins and DNA, especially transcription factors [69]. For instance, the inability of affected phosphatases to regulate kinase-mediated transduction pathways can lead to alterations of physiological functions implying in aberrant cellular growth [70]. Additionally, ROS can cause epigenetic changes, in particular, alterations in DNA methylation and histone acetylation patterns, affecting protein expression. In fact, a number of tumor suppressor genes (e.g., p15INK4B and p16INK4A) can be silenced by oxidative-induced aberrant CpG island promoter methylation [71, 72].

The deregulation of cell signaling in the early phases of carcinogenesis can trigger a wide panel of changes in cellular behaviors, which include reversible cell cycle arrest and repair, cellular senescence, and cell death [73, 74]. In many cancer types, ROS can induce the downregulation of JNK phosphatases that lead to the hyperphosphorylation of JNK and the activation of transcription factor AP-1 that enhance cell proliferation [36]. AP-1 protein activation may also participate in malignant transformation by interacting with oncogenes, as shown for H-Ras [75]. The recent studies revealed that RAS-driven proliferation requires ROS to buffer RAS-activated ERK1/2 activity [76]. Interestingly, the Nrf2 antioxidant pathway may enhance oncogenesis and avoid cellular apoptosis by counterbalancing a highly oxidative cellular environment [77]. In cancer-related inflammation, such as occurs in the gastrointestinal tract and liver cancers, ROS are known to induce NF-*κ*B signaling, an important transcription factor that upregulates several genes involved in cell transformation, proliferation, and angiogenesis, leading to the development and/or progression of cancer [78].

While ROS play a key role in maintaining mitogenic signals to drive cancer cell proliferation, they are also involved in adaptations to the metabolic stress that occurs when highly proliferative tumors outstrip their blood supply [79]. ROS generated in the hypoxic environment can prevent the hydroxylation (and thus the degradation by the ubiquitin-proteasome system) of the transcription factor HIF-1*α*, which allows its translocation to the nucleus, where it dimerizes with HIF-1*β* and promotes the transcription of genes related to proliferation, survival, and angiogenesis, such as VEGF [80]. Some tumors derived from epithelial cells upregulate not only VEGF and VEGF receptors but also matrix metalloproteinase activity through NOX1-generated ROS [81]. Importantly, several proteins related to proliferative pathways such as RAS, AKT, and ERK are also associated with cytoskeleton reorganization and cell migratory ability through pathways that can be modulated by the cell redox status [82].

## 4. Redox Homeostasis and Thyroid Carcinogenesis

Thyroid cancer corresponds to ~2.1% of all cancer diagnoses worldwide and is the eleventh most common cancer in the USA [83]. During the last decades, the incidence of thyroid cancer has increased substantially in several geographic areas in comparison with other human cancers [84]. Thyroid tumors can be derived from the follicular cells or the C cells. Approximately 95% of thyroid carcinomas are derived from the follicular thyroid cells, and the classification of thyroid cancers is done according to clinical and histological criteria [85].

In contrast to the relatively high frequency of tumors, thyroid tissue has a discrete proliferative rate. It is estimated that the human thyrocyte is quiescent for about 8.5 years, which means that each cell divides only about 5 times during adulthood [86]. On the other hand, its metabolism produces abundant amounts of H_2_O_2_. The thyroid gland is the only endocrine organ that requires H_2_O_2_ for hormone biosynthesis, which might result in a prominent mutagenic environment [87]. Quantitatively, a thyrocyte under stimulation generates almost as much H_2_O_2_ as an activated leukocyte; however, while the leukocyte dies a few hours after its activation, the lifespan of a thyrocyte is longer, allowing the accumulation of damages and thus the advent of mutations [88, 89].

As mentioned above, oxidative stress can promote DNA damage, which in turn may trigger mutations that drive tumor initiation. Maier et al. demonstrated that the normal thyroid gland has a spontaneous mutation rate (SMR) strikingly high when compared to the liver, using a rodent model. Moreover, increased levels of 8-oxoguanine (8-oxoG) immunostaining in the thyroid were also observed in relation to other organs. Elevated levels of oxidized purines and pyrimidines were found in the thyroid, and more intense 8-oxoG staining was found in epithelial cells around the lumen, precisely where DUOX2 enzyme generates H_2_O_2_ for TH biosynthesis [90]. In this context, another study with human thyroid tissue samples from follicular adenomas and carcinomas revealed increased nuclear and cytosolic levels of 8-oxoG immunoreactivity compared with nontumoral tissues [91]. Despite the fact that single DNA lesions are usually subject to an efficient repair, oxidative clustered DNA lesions (OCDLs) represent a challenge for repair systems and the possible failure of DNA repair can result in DNA double-strand breaks [92]. The incubation of a rat thyroid cell line (PCCL3) with nonlethal doses of H_2_O_2_ induced single- and double-strand breaks in DNA, as well as the phosphorylation of H_2_AX histone, compromising the genomic stability of these cells [93]. All these studies emphasize the prooxidative and consequently mutagenic and carcinogenic microenvironment that thyroid cells are exposed to during their lives.

As part of the thyroid gland physiology, the DUOX enzymes that are localized at the apical membrane of thyrocytes represent the main source of H_2_O_2_ in this tissue. Interestingly, transgenic mice with constitutive activation of the Gq-phospholipase C-Ca^2+^-PKC pathway in conjunction with the Gs-cAMP-PKA pathway seemed to cooperate with the development of malignant nodules in the thyroid gland, probably due to the activation of H_2_O_2_ production [94]. Using a heterologous expression system, we previously demonstrated that DUOX-derived H_2_O_2_ is able to oxidize TPO, inhibiting its activity [95]. Indeed, higher amounts of H_2_O_2_, at least in part produced by DUOX along with less consumption by TPO, would result in ROS accumulation [96]. However, more recent studies performed in established thyroid cancer tissues have shown no significant differences in DUOX and TPO expression and activity or even a reduced DUOX activity in comparison with normal tissue [97, 98]. Thus, the data presented in the literature seem to be variable, and a solid role of DUOX enzymes in thyroid carcinogenesis requires more investigation.

Ionizing radiation, a well-known risk factor for thyroid cancer, was recently shown to exert its effects in part through DUOX1-derived H_2_O_2_. It was demonstrated that exposure of human thyroid cells to ionizing radiation upregulates DUOX1 and its partner DUOXA1 few days after cell treatment. DUOX1-derived H_2_O_2_ induced long-term persistence of radiation-induced DNA damage, and it was associated with its own upregulation by continuous activation of the p38 MAPK signaling pathway [99]. In fact, there are accumulating evidence that ROS may act via bystander effect to disseminate stressful late effects arising from radiation exposure to nonirradiated cells in various cell types [100].

Thyrocytes also express another member of the NOX family: NOX4. As well as DUOXs, NOX4 expression and activity are positively regulated by TSH, although it seems not to participate in TH biosynthesis [101]. Differently from DUOXs, NOX4 is constitutively active and generates ROS not only at the plasma membrane but also in intracellular compartments, such as mitochondria, endoplasmic reticulum, and the nucleus [102–104]. The proximity of NOX4 to DNA in the nuclear region suggests a role for this enzyme in redox signaling in the nucleus where ROS could regulate gene expression, DNA replication, and DNA damage response. However, it is plausible to infer that NOX4 overactivity could also threaten DNA integrity and stability enabling malignant transformation. Interestingly, it has been shown that thyroid tumors express higher levels of NOX4 and its partner p22phox than nontumoral tissues, suggesting a role for this enzyme in thyroid tumorigenesis and/or tumor progression [101].

Oncogene activation can trigger DNA damage and consequently cellular senescence [105]. *BRAF* and *RAS* point mutations and *RET* gene fusions, which induce constitutive activation of the MAPK kinase signaling pathway, are the most prevalent activated oncogenes found in papillary thyroid cancer (PTC) [106]. These are driver mutations of thyroid tumorigenesis, and ROS involvement seems to be crucial [107–109]. It was reported that H_2_O_2_ exposure induced RET/PTC rearrangement in a nontumoral thyroid cell line, which was abolished by catalase [110]. Moreover, in a model of conditional expression of the oncogene H-RAS^V12^ in human thyroid cells, Weyemi et al. demonstrated the upregulation of NOX4 expression and activity, which mediated DNA damage and senescence, proving a harmful role for ROS-derived NOX4 [111]. More recently, it was shown that NOX4 is also upregulated by BRAF^V600E^ mutation in a TGF-*β*/Smad3-dependent pathway in thyroid cancer cells and that NOX4-derived ROS play a critical role in NIS repression induced by the oncogene [112]. These studies corroborate the concept that oxidative stress might be an early event in thyroid cell carcinogenesis and higher NOX4 expression seems to be an underlying mechanism.

Finally, it is important to note that a compensatory mechanism characterized by higher antioxidant defenses in response to increased ROS seems to exist in the thyroid [113]. In human thyrocyte primary culture, an augmented expression of antioxidant genes was noticed after exposure to H_2_O_2_ and increased DNA damage was detected after experimental depletion of GSH content [114]. These findings indicate that impairment of detoxification systems might also support the detrimental effect of high H_2_O_2_ levels in the thyroid.

## 5. Estrogens and Redox Homeostasis in Thyroid Carcinogenesis

Estrogens are steroid hormones related to a broad spectrum of physiological functions, extending from the regulation of the menstrual cycle and reproduction to modulation of bone density and brain and cardiovascular functions, as well as cholesterol homeostasis [115]. The most active and potent estrogen is estradiol, which is secreted primarily by the ovaries and in lesser quantities by the adrenal gland [116]. Biological effects mediated by estradiol in target tissues primarily occur due to its binding to specific intracellular receptors, estrogen receptor *α* (ER*α*) and *β* (ER*β*), which are members of a large family of nuclear transcription factors. Conformational changes allow receptor dimerization in the presence of estradiol, translocation to the nucleus, and the binding of the estrogen-ER complex to the estrogen response element (ERE) located in or near the promoter region of the target genes [117]. Alternatively, estrogen may exert rapid effects through intracellular noncanonical signaling pathways, which are independent of gene transcription. The membrane-associated estrogen receptor (mER), the orphan member of the G protein-coupled receptor superfamily GPER-1 (GPR30), and another membrane-bound ER, referred as ER-X, have been reported to act independently of the classical intracellular ERs, triggering effects ranging from growth and proliferation to survival and development [118–120]. Indeed, mainly due to its proliferative and antiapoptotic effects, estrogen is recognized as a well-established risk factor for a variety of cancers, such as breast and endometrium [121].

Although a variety of studies on ER expression have been performed in both normal and neoplastic thyroid tissues with extremely heterogeneous results, the first demonstration of a direct growth-stimulatory effect of estrogen was shown in the differentiated rat thyroid cell FRTL-5. This cell line expresses functional ER*α*, and E2 stimulation enhanced DNA synthesis and proliferation [122]. Sequentially, several lines of evidence demonstrated that E2 induces cell growth in primary cultures of human thyrocytes obtained from benign and malignant thyroid nodules and in most human thyroid carcinoma cell lines [123–126]. An inverse relationship between ER*α* and ER*β* expression has also been reported in human thyroid cancer cells [127, 128]. A proliferative and antiapoptotic effect together with a role in the metastasis process has been related to ER*α*, whereas ER*β* seems to induce differentiation and proapoptotic effects [129]. Moreover, evidence from clinical studies in thyroid cancers strongly suggests an association between the presence of ER*α* expression and partial or total lack of ER*β* expression with more aggressive behavior or a trend towards the presence of local metastases at diagnosis [130–132]. In thyroid cancer cell lines, the proliferative effects of estradiol seem to be mediated through the regulation of genes involved in growth control, such as bcl-2, Bax, c-fos, E-cadherin, and vimentin [133, 134]. It is well documented that E2 amplifies its own growth-promoting effect by upregulating ER*α* expression in thyroid carcinoma cells [123, 133]. In addition, nongenomic actions of E2, mainly through the activation of ERK1/2 and PI3K/Akt signaling pathways, are known to play a pivotal role in thyroid tumorigenesis [126]. In mice, it has been proposed that E2 increases the susceptibility of females to thyroid follicular carcinomas through PI3K pathway activation and p27 inhibition [135]. Collectively, these clinical and experimental data support a relevant role of estrogen and its receptors in the pathogenesis and even progression of thyroid cancer; however, the mechanisms involved in E2 thyroid action remain elusive.

In the last decade, special attention has been given to the relationship between estrogen metabolism and thyroid cancer. Some authors have hypothesized that estrogens can become endogenous carcinogens based on the discovery that specific reactive estrogen metabolites (catechol estrogen quinones) can react with DNA and promote mutations in critical genes leading to the initiation of cancer [136]. Indeed, estrogens are metabolized via two major pathways that lead to the formation of 16*α*-OHE1 (E2) or the catechol estrogens 2-OHE1 (E2) and 4-OHE1 (E2). When the mechanisms of catechol inactivation are not efficient, oxidation of the catechol estrogens to semiquinones (SQ) and then quinones (Q), catalyzed by cytochrome P450 (CYP) or peroxidase, can occur. Oxidation of semiquinones to quinones can also be performed by molecular oxygen, and the reduction of estrogen quinones to semiquinones by CYP reductase terminates the redox cycle. In this process, several types of ROS can be generated, and as discussed above, increased availability of ROS per se already represents a potential initial step for cancer initiation. The formation of E1 (E2)-3,4-Q and E1 (E2)-2,3-Q can be neutralized by glutathione (GSH) or by the reduction to their respective catechols by quinone reductase. If not, they can react with DNA to form predominantly the depurinating adducts: 4-OHE1 (E2)-1-N3Ade plus 4-OHE1 (E2)-1-N7Gua (97%) from E1 (E2)-3,4-Q and 2-OHE1 (E2)-6-N3Ade (3%) from E1 (E2)-2,3-Q. Depurinating adducts are closely associated with the generation of the apurinic sites in the DNA, and errors in the repair of these sites can induce critical mutations favoring the initiation of many common types of human cancer. Studies in rodent models treated with E2-3,4-Q have shown a correlation between the sites of the formation of depurinating DNA adducts and H-RAS mutations in skin and mammary glands [137, 138]. Concerning the thyroid, a case-control study utilizing the urine sample was conducted with women diagnosed with thyroid cancer and healthy women as the control. Thirty-eight estrogen metabolites, conjugates, and DNA adducts were analyzed by ultraperformance liquid chromatography/tandem mass spectrometry, and the ratio of adducts to metabolites and conjugates was significantly higher in the cancer group compared to the control [139]. The authors suggest that the formation of these adducts could be a causative factor in the etiology of several cancers, but more investigations are necessary.

Our group has proposed another mechanism through which estradiol regulates ROS generation in the thyroid gland. We have detected higher H_2_O_2_ production and NOX4 expression in the thyroids of adult female rats in comparison with their male counterparts under physiological conditions [140]. This gender disparity was not found in prepubertal animals, in which serum E2 levels are low, indicating a possible direct role of this hormone in the regulation of NOX4. Consistent with this hypothesis, monitoring the estrous cycle of rats, we observed that in the proestrus phase, which is characterized by an estrogen peak, the levels of NOX4 mRNA were increased in comparison to the other phases and higher production of H_2_O_2_ was detected in the estrus phase. Additionally, catalase expression and activity, together with the levels of free thiol groups, were lower in the thyroid of adult females compared with males. In an *in vitro* approach, 17*β*-estradiol treatment was able to increase H_2_O_2_ generation and NOX4 expression in the normal rat thyroid cell line (PCCL3), suggesting a crucial role of this hormone in the sexual dimorphism found in thyroid redox homeostasis [140]. These results point to NOX4 as a putative target of estrogen action in thyroid tissue, which might be involved in the higher susceptibility to thyroid cancer that is observed in women (Figure 2).

As cited above, the wide range of ROS effects can vary depending on the specific stage of carcinogenesis. Both estrogen and ROS have been shown to participate in the induction and maintenance of proliferative stimulus in several cell types. In the thyroid context, it was demonstrated that ER*α* contributes to thyroid tumorigenesis not only by stimulating cell proliferation but also by enhancing autophagy, an important prosurvival catabolic process, through ERK1/2-related pathways and ROS-dependent manner [141]. Furthermore, in thyroid cancer cell lines, mitochondria are also sources of ROS in response to estrogen, which was associated with UCP2 downregulation [142]. Both ERs (*α* and *β*) are expressed in mitochondria, and estrogen response element- (ERE-) like sequences are present in the mitochondrial genome together with estrogen-binding proteins (EBPs) [143–146], but were not shown in the thyroid.

Ultimately, it is worth to note that VEGF is upregulated by estrogen in the thyroid gland, and that the thyroid weight and mean vascular area were shown to be lower in ovariectomized rats in comparison with ovariectomized rats treated with estrogen [147]. In this regard, it was demonstrated that an increase in intracellular ROS elicited stabilization of HIF-1*α* and VEGF release, but simultaneous treatment with the antioxidant N-acetylcysteine abrogated these effects [148]. HIF-1*α* is overexpressed in thyroid cancer [149]; it is thus tempting to speculate the existence of a possible crosstalk among estrogens, ROS, and VEGF during thyroid tumor progression.

## 6. Conclusions

In this review, we propose that the sexual dimorphism found in thyroid cancer can be related to an important relationship between ROS modulation and estradiol action. Physiologically, the thyroid gland is exposed to considerably high amounts of H_2_O_2_, which might act as a potent mutation-driver agent through the induction of genomic instability. The female thyroid gland seems to be exposed to greater amounts of H_2_O_2_ than male thyroids, at least in rodents. In face of the strong evidence of estrogen actions in the thyroid and its ability to regulate ROS generation, it is conceivable to believe that the higher susceptibility of thyroid cancer in women could be due, at least in part, to higher ROS levels and the consequent accumulation of oxidative DNA damage. NOX4 seems to be the source of estrogen-upregulated ROS in thyrocytes. However, the precise localization of NOX4 in the thyroid cell is yet to be defined. A more in-depth mechanistic investigation of the molecular events that underlie this working hypothesis is essential for a better understanding of the process of thyroid carcinogenesis.

## Figures and Tables

**Figure 1:** The main events in the tumorigenesis process triggered by different levels of oxidative stress. The initiation stage is associated with low oxidative stress, which leads to the activation of Nrf2 (nuclear factor erythroid 2-related factor 2) that in turn induces the expression of a set of antioxidant genes, as an example of the stress response. In addition, oxidation of DNA may cause oxidative damages that culminate in genomic instability. These events provide the deregulation of crucial signaling pathways. In the promotion stage, intermediate levels of ROS are involved in the activation of key transcription factors, such as NF-*κ*B and AP-1, and also in the inhibition of phosphatases that promote cell survival and proliferation. This stage is already marked by extensive damage of lipids, proteins, and nucleic acids. Concerning the progression stage, the high levels of ROS produced by cancer cells are related to HIF-1*α* stabilization that enables angiogenesis and the activation of metalloproteinases that support the extracellular matrix (ECM) remodeling.

**Figure 2:** Proposed model of estrogen-induced ROS generation increase in thyrocyte. Estradiol stimulates ROS production by NOX4 that is possibly located in the plasma membrane, endoplasmic reticulum, nuclear membrane, and mitochondria, as well as generates ROS through its own metabolization. ROS can reach the nucleus and promote several alterations that might contribute to thyroid carcinogenesis. Estrogen metabolization pathway also gives rise to the mutagenic DNA depurinating adducts. It is important to point out that the intracellular increase of ROS in response to estrogen can also positively modulate important carcinogenesis-related signaling pathways, such as ERK1/2 and PI3K/Akt. DSB: double-strand break; DUOX: dual oxidase; E2: estrogen; NOX4: NAPDH oxidase 4; ROS: reactive oxygen species; SSB: single-strand break; TPO: thyroperoxidase.
